RETRACTED

# Silencing CircHIPK3 Sponges miR-93-5p to Inhibit the Activation of Rac1/PI3K/AKT Pathway and Improves Myocardial Infarction-Induced Cardiac Dysfunction

**DOI:** 10.3389/fcvm.2021.645378

**Published:** 2021-04-30

**Authors:** Yijin Wu, Min Wu, Jue Yang, Ying Li, Wenying Peng, Meifen Wu, Changjiang Yu, Miaoxian Fang

**Affiliations:** ^1^Department of Intensive Care Unit of Cardiac Surgery, Guangdong Provincial People's Hospital, Guangdong Academy of Medical Sciences, Guangdong Cardiovascular Institute, Guangzhou, China; ^2^Department of Cardiac Surgery, Guangdong Provincial People's Hospital, Guangdong Academy of Medical Sciences, Guangdong Cardiovascular Institute, Guangzhou, China

**Keywords:** myocardial infarction, cardiac dysfunction, circHIPK3, miR-93-5p, Rac1, PI3K/AKT pathway

## Abstract

The ceRNA network involving circular RNAs (circRNAs) is essential in the cardiovascular system. We investigated the underlying ceRNA network involving circHIPK3 in myocardial infarction (MI). After an MI model was established, cardiac function was verified, and myocardial tissue damage in mice with MI was evaluated. A hypoxia model of cardiomyocytes was used to simulate MI *in vivo*, and the expression of and targeting relationships among circHIPK3, miR-93-5p, and Rac1 were verified. The apoptosis of cardiomyocyte was identified. Gain- and loss-of-functions were performed to verify the ceRNA mechanism. The MI-modeled mice showed cardiac dysfunction and enlarged infarct size. CircHIPK3 was highly expressed in mouse and cell models of MI. Silencing circHIPK3 reduced infarct size, myocardial collagen deposition, and myocardial apoptosis rate and improved cardiac function. CircHIPK3 sponged miR-93-5p, and miR-93-5p targeted Rac1. Overexpression of miR-93-5p inhibited MI-induced cardiomyocyte injury and eliminated the harmful effect of circHIPK3. CircHIPK3 acted as ceRNA to absorb miR-93-5p, thus promoting the activation of the Rac1/PI3K/AKT pathway. We highlighted that silencing circHIPK3 can upregulate miR-93-5p and then inhibit the activation of Rac1/PI3K/Akt pathway, which can improve MI-induced cardiac dysfunction.

## Introduction

Myocardial infarction (MI) is among the most serious health threats, which leads to dysfunction and irreversible loss of cardiomyocytes (1). MI ruins the viable myocardium, resulting in cardiac dysfunction and increased risk of heart failure (2). Upon MI, massive cardiomyocyte death triggers a strong inflammatory response, which is a vital process of cardiac injury, repair, and remodeling (3). Patients with MI are often affected by psychological disorders such as depression, anxiety, and post-traumatic stress disorder (4). About 5% of patients with MI suffer from cardiogenic shock as a complication, with a mortality of ≥30% (5). After an episode of MI, patients remain at risk for recurrent arrhythmia, heart failure, and sudden death (6). The ability of cardiac tissue to recover after MI is affected by numerous complex cellular and molecular pathways (7). Despite decades of therapeutic advances, MI remains a leading cause of death (8). In such a context, it is urgent to search for effective molecular pathways to provide insight into the prevention and management of MI.

RETRACTED

Circular RNAs (circRNAs) have been defined as naturally occurring RNAs mainly engaged in regulating gene expression (9, 10). In the cardiovascular system, circRNAs significantly mediate important physiological and pathological processes (11). Using circRNA microarray assays, Wu et al. have reported many differentially expressed circRNAs in murine left ventricular tissues with MI-induced heart failure (12). CircHIPK3 is widely expressed in diverse diseases, such as preeclampsia, diabetes, osteoblasts, and retinal vascular dysfunction (13). CircRNAs are implicated in various biological functions by interacting with proteins and absorbing microRNAs (miRs) (14). miRs are frequently dysregulated in vascular diseases, such as limb ischemia and MI (15). For instance, circHIPK3 worsens myocardial ischemia–reperfusion (I/R) injury by sponging miR-124-3p (16). Exosomal circHIPK3 secreted from hypoxic cardiomyocytes monitors oxidative damage in cardiac microvascular endothelial cells through the miR-29a/IGF-1 axis (17). Hence, we speculated that circHIPK3 may regulate cell behavior in MI *via* interacting with miR to form a circRNA–miR–mRNA network. Consequently, we performed a series of histological and molecular experiments to identify the circRNA–miR–mRNA network and to study the underlying molecular mechanism, with the purpose to provide some novel therapies against MI.

## Methods

### Ethics Statement

This study was supervised and approved by the ethics committee of Guangdong Provincial People's Hospital, Guangdong Academy of Medical Sciences, Guangdong Cardiovascular Institute. All participants signed the informed consent. This study conformed to all relevant ethical norms of research involving human participants.

### Establishment of MI Mouse Model

A total of 70 male C57BL/6J mice at specific pathogen-free (SPF) grade (8–11 weeks old, 20.22 ± 1.46 g) were obtained from Hunan SJA Laboratory Animal Co., Ltd. (Changsha, Hunan, China). Ten mice were randomly selected as normal group, and the remaining 60 mice were used to construct the MI model. All mice were fed in a SPF animal laboratory and given normal diet with humidity of 60–65% at 22–25°C. Before modeling, mice in each group were anesthetized by intraperitoneal injection of 0.05 mg/g pentobarbital sodium (P3761, Sigma-Aldrich, Merck KGaA, Darmstadt, Germany). The left descending coronary artery (2 mm below the left atrioventricular junction) was ligated with 7–0 suture to establish the MI model. In the sham group, the other steps were the same as detailed above except ligation. After the surgery, the thoracic cavity was closed, and the survival and wound infection of mice were monitored. Samples were collected 28 days after the surgery. The mice were anesthetized when the samples were collected, and then the thoracic cavity was opened to isolate the mouse heart. Each group of adenovirus vector (1 × 10^9^ pfu/mouse, Genepharma, Suzhou, China) was injected into MI-molded C57BL/6 mice *via* the tail vein. The sh-CircHIPK3 and negative control shRNA (sh-NC) were designed and purchased from Invitrogen (CA, USA). The recombinant adenovirus vector carrying sh-CircHIPK3 was constructed by inserting the constructed vector into the adenovirus vector pAd-PPARGC1A. The ascending aorta was clipped for adenovirus transfection. The left ventricle was injected with 70 μl (108 TU/xml) plasmid carrying sh-CircHIPK3 or sh-NC. After 15 s of temporary occlusion of the aorta, the plasmid was forced into the coronary artery. The sham-operated mice were treated with 70 μl Dulbecco's modified Eagle's medium (DMEM). At 4 weeks after adenovirus injection, transthoracic echocardiography was performed (18, 19).

RETRACTED

### Cardiac Function Detection

Cardiac function was assessed using echocardiography in small animals (Vevo 2100, Visualsonics, Toronto, Canada) to test left ventricular end diastolic diameter (LVEDd), left ventricular end systolic diameter (LVESD), left ventricular short axis ejection fraction (EF), and fraction shortening (FS). EF (%) = [(EDD^3^ – ESD^3^)/EDD^3^] × 100; FS (%) = [(LVEDd – LVESD)/LVEDd] × 100. Six consecutive cardiac cycles were measured in the same animal. The animals were blindly selected (20–22).

### 2,3,5-Triphenyltetrazolium Chloride Staining

Left ventricular apical tissue was randomly extracted from mice in each group. Ultrathin sections (50–60 nm) were cut along the long axis of the left ventricle with a vibrator. Left ventricular wall myocardium was stained with 1% 2,3,5-triphenyltetrazolium chloride (TTC; batch number: 71016588, Sinopharm Chemical Reagent Co, Ltd. Shanghai, China) to observe the ultrastructure. Sections were stained in 1% tricalcium phosphate buffer solution (CAS No. 2530-85-0; Guidechem Shanghai, China). The infarcted myocardium was gray white, and the viable myocardium was in normal color. The infarcted myocardium was separated from the viable myocardium. The images of each part were taken with a camera (Leica digital camera 480; Leica Microsystems, GmbH, Wetzlar, Germany), and the MI area was measured by ImageJ 1.26 image analysis software (National Institutes of Health, Bethesda, MD, USA): MI area (mm^2^) = MI area (mm^2^)/total left ventricular area (mm^2^) ×100% (23).

RETRACTED

### Masson Staining

After dewaxing and dehydration, the sections were dyed with ponceau S dye for 2 min and treated in 0.2% glacial acetic acid solution for 2 min and 5% molybdic acid solution for 2 min. Next, the sections were washed in 0.2% glacial acetic acid solution for 2 min, stained with methyl green staining for 3 min, washed with water, color-separated with 95% ethanol, dehydrated with ethanol, cleared with xylene, and sealed with neutral gum. Under an optical microscope (×100), the area rich in collagen fibers was stained blue, and the cell matrix was stained red. Ten visual fields were selected from each section randomly. The images were obtained and analyzed by ImageJ analysis software. The degree of liver fibrosis was expressed by the percentage of fibrosis area in the whole area.

### TUNEL Staining

Frozen sections of mouse myocardium were incubated for 5 min with phosphate-buffered saline (PBS) containing 0.1% Triton X-100. In the following steps, as described in the instructions of a TUNEL kit (C1090, Beyotime, Shanghai, China), the TUNEL detection solution was prepared according to the volume ratio of TdT enzyme and fluorescent labeling solution 1:9 and fully mixed. The cell surface was washed with PBS once, and 50 μl TUNEL detection solution was added to each sample. They were incubated at 37°C for 60 min. Then, the staining solution was removed, and sections were washed with PBS three times. The surface was dripped with anti-fluorescence quenching sealing and observed by a fluorescence microscope (Leica SR, GSD, Leica).

### Establishment of Hypoxia Model of Cardiomyocytes

HL-1 cells were cultured with DMEM (Gibco, Thermo Fisher, Waltham, Ma, USA) containing 10% fetal bovine serum (Excell Bio, Genetimes, Shanghai, China), 100 U/ml penicillin, and 100 μg/ml streptomycin at 37°C with 5% CO_2_ and saturated humidity. A hypoxia model was established 72 h after transfection. The model cells was cultured in hypoxia (Hypo group), namely, 93% N_2_, 2% O_2_, and 5% CO_2_. The control cells were cultured under normal conditions. After 24 h of culture, the following tests were carried out (24, 25).

### RNA Fluorescence *in situ* Hybridization

FISH assay was applied to examine the localization of circHIPK3 in cardiomyocytes. According to the Ribo^TM^ lncRNA FISH Probe Mix (Red) (Guangzhou Ribo Biotechnology Co., Ltd., Guangzhou, China), circHIPK3 probe was designed, and the cardiomyocytes were seeded into six-well plates with a cover glass. The confluence was about 80% after 1 day of culture. After cleaning with PBS, the glass was fixed with 1 ml 4% paraformaldehyde and detached with protease K (2 μg/ml), glycine, and acetophthalein reagent, followed by 1-h incubation with prehybridization solution (250 μl) at 42°C. The prehybridized solution was aspirated, and 250 μl of hybridization solution containing probe (300 ng/ml) was added and hybridized overnight at 42°C. After three times of cleaning with PBS containing 0.05% Tween-20 (PBST), DAPI (1:800) solution diluted with PBST was supplemented to the 24-well plates for 5-min nucleus staining, following three PBST washes, each for 3 min. The slides were sealed with fluorescent mounting media, and five different fields of vision were photographed under a fluorescence microscope (Olympus, Japan) (26).

RETRACTED

### Dual-Luciferase Reporter Gene Assay

The synthesized Rac1 3′UTR gene fragment was inserted into pGL3 reporter (Promega, WI, USA) by endonuclease sites XhoI and BamHI. Complementary mutation sites of seed sequence were designed on wild-type (WT) Rac1. After restriction endonuclease digestion, the target fragment was inserted into pGL3 reporter vector by T4 DNA ligase. The constructed luciferase reporter plasmid Rac1-WT or mutant (MUT) was cotransfected with miR-93-5p mimic or mimic NC into HEK293T cells. After 48-h transfection, the cells were harvested and lysed. Luciferase activity was detected on Luminometer TD-20/20 detector (E5311, Promega, WI, USA) using dual-luciferase reporter assay system (E1910). The binding relationship between circHIPK3 and miR-93-5p was detected by the same method.

### RNA Immunoprecipitation

RNA immunoprecipitation (RIP) kit (Millipore, Billerica, MA, USA) was utilized to identify the binding of circHIPK3 with Ago2 protein. The cardiomyocytes were cleared in precooled PBS with the supernatant removed. Thereafter, the cells were lysed with the same volume of RIPA lysate in an ice bath and centrifuged for 10 min at 14,000 rpm at 4°C, and the supernatant was removed. The cardiomyocytes were cocultured with antibodies for coprecipitation. In each coprecipitation reaction system, 50 μl magnetic beads was washed and then resuspended into 100 μl RIP wash buffer and incubated with 5 μg antibody for binding. After cleaning, the magnetic beads–antibody complex was resuspended in 900 μl RIP wash buffer and incubated overnight at 4°C with 100 μl cell extract. The samples were put on a magnetic stand to obtain the bead protein complex. The samples were detached with protease K to extract RNA for subsequent detection. The antibody used was rabbit anti-Ago2 (ab186733, 1:50, Abcam, Cambridge, MA, USA) for 30 min, with rabbit anti-IgG (ab109489, 1:100) as negative control.

RETRACTED

### RNA Pull-Down Assay

Cells were transfected with 50 nM biotin-labeled WT-bio-miR-93-5p and MUT-miR-93-5p (Wuhan Genecreate Bioengineering Co., Ltd, Wuhan, Hubei, China) for 48 h. Then, cells were harvested, washed in PBS, and incubated in a specific lysis buffer (Ambion, Austin, Texas, USA). The lysate was supplemented with M-280 streptavidin magnetic beads (S3762, Sigma-Aldrich) precoated with RNase-free BSA and yeast tRNA (TRNABAK-RO, Sigma-Aldrich) overnight at 4°C. The samples were washed twice with precooled lysis buffer, three times with low salt buffer, and once with high salt buffer. The binding RNA was purified by TRIzol, and the enrichment of circHIPK3 was measured by reverse transcription quantitative polymerase chain reaction (RT-qPCR).

### RT-qPCR

Total RNA was extracted by TRIzol (Invitrogen). According to the instructions, the first-strand cDNA synthesis kit (Takara, Japan) was used for reverse transcription to synthesize the first-strand cDNA. Gene expression was detected by real-time qPCR using SYBR Premix Ex Taq kit (Takara, Japan). The PCR reaction conditions were pre-denaturation at 95°C for 10 min and 40 cycles of 94°C for 30 s, 59°C for 30 s, and 72°C for 30 s on ABI Prism 7500 Fast Real-Time PCR system (Applied Biosystems, MA, USA). Gene expression was calculated by 2^−Δ*ΔCT*^ method, with U6 or GAPDH as an internal reference. The primer sequences are displayed in Table 1. When detecting RNA in mouse myocardial tissue samples, 0.1 g tissue sample was ground with a grinder (KZ-II, Servicebio, Wuhan, China) at 4°C, and then extract RNA was extracted with Trizol.

**Table 1:** Primer sequences for RT-qPCR.

**Gene**	**Sequence**
CircHIPK3	F: 5′-TAGACTTTGGGTCGGCCAGT-3′
	R: 5′-TGGAATACACAACTGCTTGGC-3′
miR-93-5p	F: 5′-AAGTGCTGTTCGTGCAGGT-3′
	R: 5′-CTCGGGAAGTGTAGCTCA-3′
Rac1	F: 5′-GTAAAACCTGCCTGCCTGCTCATCA-3′
	R: 5′-GGACGCAATCTGTCATAATCTTC-3′
GAPDH	F: 5′-AGTGCCAGCCTCGTCTCATA-3′
	R: 5′-GGTAACCAGGCGTCCGATAC-3′
U6	F: 5′-CTCGCTTCGGCAGCACA-3′
	R: 5′-AACGCTTCACGAATTTGCGT-3′

### Western Blot

Total protein was extracted by RIPA (R0010, Solarbio, Beijing, China). The transfected cells were washed three times with 1 × PBS. An appropriate amount of protein lysates was added into each cell bottle, collected in EP tube, and left standing on ice for 30 min. The sample was centrifuged for 10 min at 4°C, 13,000 × *g*, and the supernatant was collected and placed in an ice box. The protein concentration was quantified by bicinchoninic acid kit (P0011, Beyotime). The proteins were separated by polyacrylamide gel electrophoresis and transferred to 0.2 μm polyvinylidene fluoride membranes (ISEQ10100, Millipore). Then, the membranes were blocked using tris-buffered saline containing 0.1% Tween-20 (TBST) with 5% skim milk powder (D8340, Solarbio) on a decolorizing shaker for 1 h. TBST solution containing 1% skim milk powder diluted the antibody as the primary antibody diluent. The membranes were added with the primary antibody diluent at 4°C overnight. On the next day, the membranes were washed by TBST three times, each time for 10 min on a decolorizing shaker. The horseradish peroxidase-labeled goat anti-rabbit IgG antibody (1:5,000, A0208, Beyotime) was diluted with TBST solution containing 1% skim milk powder as the diluent of secondary antibody and incubated for 1 h. The membranes were washed three times by TBST, each time for 10 min on the decolorizing shaker. Digital chemiluminescence (C-DiGit® Blot Scanner Li-Cor, NE, USA) was used for detection, and ImageJ was used for analysis. With GAPDH as the internal reference, the ratio of gray value of target band to GAPDH band was used as the relative protein level. The primary antibodies included rabbit anti-Bax (ab32503; 1:2,000), cleaved caspase-3 (ab32042; 1:500), Bcl-2 (ab32124; 1:000), p-PI3K (ab32089; 1:1,000), p-AKT (ab8805; 1:500), t-PI3K (ab70912; 1:100), t-AKT (ab179463; 1:500), and GAPDH (ab8245; 1:1,000).

RETRACTED

### Statistical Analysis

All statistical analyses were conducted using SPSS 18.0 software (IBM Corp., Armonk, NY, USA). The data in normal distribution and homogeneity of variance were expressed as mean ± standard deviation. The independent-sample *t*-test compared two groups of data in non-paired design. The comparison among multiple groups was analyzed using one-way analysis of variance (ANOVA) and Tukey's multiple-comparisons test. The correlation of circHIPK3 and miR-93-5p was analyzed using Pearson's correlation analysis. *p* < 0.05 meant that the difference was statistically significant.

## Results

### CircHIPK3 Is Highly Expressed in the Mouse Model and Cell Model of MI

CircHIPK3 can inhibit cardiomyocyte proliferation and induce cardiomyocyte apoptosis after myocardial I/R injury, which may be a promising approach of I/R (16), but its mechanism in MI needs further study. Echocardiography showed that LVEDd and LVESD increased, and EF% and FS% decreased in MI group compared with sham group (all *p* < 0.05) (Figure 1A). TTC staining showed that, relative to the sham group, the infarct size of mice in the MI group was clearly increased (*p* < 0.05) (Figure 1B). These results indicate that the model of MI in mice was successfully established.

RETRACTED

**Figure 1:** CircHIPK3 is highly expressed in the mouse model and cell model of myocardial infarction (MI). **(A)** Echocardiography was used to detect the changes of cardiac function-related indexes after modeling, *n* = 10. **(B)** 2,3,5-Triphenyltetrazolium chloride staining was used to detect the infarct area, *n* = 10. **(C)** TUNEL staining was used to detect apoptosis after MI *in vitro*. **(D)** RT-qPCR was used to detect the expression of CircHIPK3 in myocardial tissue of MI mice and *in vitro* cell model. The value in the figures is the measurement data, which is expressed as mean ± standard deviation. The comparison between two groups was analyzed by independent-sample *t*-test. *compared with sham group, *p* < 0.05; ^#^compared with control group, *p* < 0.05. The experiment was repeated three times.

In this study, cardiomyocytes were treated with hypoxia to simulate the *in vitro* model of MI. TUNEL staining revealed that the apoptotic ability of the hypoxia group was higher than that of the control group (*p* < 0.05) (Figure 1C). Then, RT-qPCR was used to test circHIPK3 expression in the myocardial tissue of MI model mice and cell model. Compared with the sham group, circHIPK3 expression in the myocardial tissue of MI mice and cell model, respectively, was significantly increased (both *p* < 0.05) (Figure 1D).

### CircHIPK3 Downregulation Can Reduce Cardiomyocyte Apoptosis After MI and Improve Cardiac Function

From the above-mentioned results, we knew that circHIPK3 was highly expressed in myocardial tissues and cell model with MI, so we set sham group, MI group, MI + sh-NC group, MI + sh-CircHIPK3 group in mice, control group, hypoxia group, hypoxia + sh-NC group, and hypoxia + sh-CircHIPK3 group *in vitro* cardiomyocytes to examine the effects of silencing circHIPK3 on MI mice and hypoxia-induced cardiomyocyte injury.

RT-qPCR detected circHIPK3 expression in myocardial tissue and showed that, vs. the MI + sh-NC group, circHIPK3 expression in the MI + sh-CircHIPK3 group was obviously decreased (*p* < 0.05) (Figure 2A), indicating that circHIPK3 was successfully knocked down *in vivo*. TTC staining showed that, relative to the MI + sh-NC group, the infarct size of MI + sh-CircHIPK3 group was clearly decreased (*p* < 0.05) (Figure 2B). Masson staining showed that interference with circHIPK3 significantly reduced collagen deposition (*p* < 0.05) (Figure 2C). TUNEL staining showed that interference with circHIPK3 significantly reduced the rate of myocardial apoptosis (*p* < 0.05) (Figure 2D). Relative to MI + sh-NC group, the levels of Bax and cleaved caspase-3 in the MI + sh-CircHIPK3 group were obviously decreased, and Bcl-2 was elevated (all *p* < 0.05) (Figure 2E). No significant difference was observed between MI group and MI + sh-NC group (*p* > 0.05).

RETRACTED

**Figure 2:** CircHIPK3 downregulation can reduce cardiomyocyte apoptosis after myocardial infarction (MI) and improve cardiac function. **(A)** RT-qPCR detected the expression of CircHIPK3 in myocardial tissue. **(B)** 2,3,5-Triphenyltetrazolium chloride staining was used to detect infarct size. **(C)** Masson staining was used to detect collagen deposition. **(D)** TUNEL staining was used to observe the apoptosis of myocardial tissue. **(E)** The expression of Bax, cleaved caspase-3, and Bcl-2 protein, respectively, was detected by Western blot analysis. **(F)** RT-qPCR detected CircHIPK3 expression in cardiomyocytes *in vitro*. **(G)** The apoptosis of cardiomyocytes was detected by TUNEL staining. **(H)** Western blot analysis detected the expression of Bax, cleaved caspase-3, and Bcl-2 protein. The value in the figures is the measurement data, which is expressed as mean ± standard deviation. The comparison among multiple groups was analyzed by one-way ANOVA, followed by Tukey's multiple-comparisons test. *compared with sham group, *p* < 0.05; ^#^compared with MI + sh-NC group, *p* < 0.05; ^&^compared with control group, *p* < 0.05; ^@^compared with hypoxia + sh-NC group, *p* < 0.05. The experiment was repeated three times.

RT-qPCR detected circHIPK3 expression in cardiomyocytes *in vitro*. Compared with the hypoxia + sh-NC group, circHIPK3 expression in the hypoxia + sh-CircHIPK3 group was significantly decreased (*p* < 0.05) (Figure 2F), indicating that circHIPK3 was successfully interfered with *in vitro*. TUNEL staining showed that, compared with hypoxia + sh-NC group, cardiomyocyte apoptosis in hypoxia + sh-CircHIPK3 group was significantly decreased (*p* < 0.05) (Figure 2G). The levels of Bax and cleaved caspase-3 were clearly decreased, and Bcl-2 expression was raised in cardiomyocytes (all *p* < 0.05) (Figure 2H).

The above-mentioned results of animal experiments and cell experiments showed that interference with circHIPK3 can reduce cardiomyocyte apoptosis after MI and improve cardiac function.

### CircHIPK3 Sponges miR-93-5p as a ceRNA

To explore the mechanism of circHIPK3, we first detected the expression and localization of CircHIPK3 by RNA-FISH. The result displayed that circHIPK3 was mainly expressed in the cytoplasm (Figure 3A). Through the Starbase website (http://starbase.sysu.edu.cn/agoClipRNA.php?source=mRNA), we confirmed that circHIPK3 bound to miR-93-5p (Figure 3B). Dual-luciferase assay exhibited that the luciferase signal of WT-CircHIPK3 in miR-93-5p mimic transfection group was lower than that in mimic NC group. However, the luciferase activity of mutant 3′UTR was not obviously different (*p* > 0.05) (Figure 3C). The specific adsorption level of circHIPK3 to Ago2 was higher than that of IgG group (*p* < 0.05) (Figure 3D). RNA pull-down verified that the enrichment level of circHIPK3 in Bio-miR-93-5p-WT group was higher than that in Bio-probe NC group (*p* < 0.05), but it did not significantly differ in Bio-miR-93-5p-MUT group (Figure 3E). These results suggested that circHIPK3 acting as a ceRNA absorbed miR-93-5p, thus affecting miR-93-5p expression.

RETRACTED

**Figure 3:** CircHIPK3 sponges miR-93-5p as a ceRNA. **(A)** RNA-FISH was used to detect the subcellular localization of CircHIPK3. **(B)** Bioinformatic website predicted the binding relationship between CircHIPK3 and miR-93-5p. **(C)** Dual-luciferase reporter gene assay was used to verify the binding relationship between CircHIPK3 and miR-93-5p. **(D)** RIP assay was used to detect the relationship between CircHIPK3 and Ago2. **(E)** RNA pull-down test was used to verify the binding of CircHIPK3 and miR-93-5p. The value in the figures is the measurement data, which is expressed as mean ± standard deviation. The comparison between two groups was analyzed by independent-sample *t*-test. The comparison among multiple groups was analyzed by one-way ANOVA, followed by Tukey's multiple-comparisons test, *p < 0.05. The experiment was repeated three times.

### Overexpression of miR-93-5p Reverses the MI-Induced Myocardial Injury Stimulated by CircHIPK3

Then, we shifted to investigating the expression profile and role of miR-93-5p in MI models. RT-qPCR detected miR-93-5p expression in myocardial tissue and demonstrated that miR-93-5p expression in myocardial tissue of MI group was lower than that of sham group (*p* < 0.05) (Figure 4A), and Pearson's correlation analysis showed that miR-93-5p expression was negatively correlated with circHIPK3 (*p* < 0.05) (Figure 4B). To further study whether circHIPK3 exerts functions through miR-93-5p, we set up oe-NC + agomiR-NC group, oe-CircHIPK3 + agomiR-NC group, and oe-CircHIPK3 + miR-93-5p agomiR cotransfection group. TTC staining showed that, compared with oe-NC + agomiR-NC group, the infarct size of oe-CircHIPK3 + agomiR-NC group was significantly increased (*p* < 0.05), while compared with oe-CircHIPK3 + agomiR-NC group, the infarct area of oe-CircHIPK3 + miR-93-5p agomiR group was significantly decreased (all *p* < 0.05) (Figure 4C). Masson staining showed that overexpression of circHIPK3 and miR-93-5p at the same time significantly reduced collagen deposition in myocardial tissue compared with overexpression of circHIPK3 alone (*p* < 0.05) (Figure 4D). TUNEL staining presented that, compared with oe-NC + agomiR NC group, the apoptosis rate of myocardial tissue in oe-CircHIPK3 + agomiR-NC group was clearly increased (*p* < 0.05), while compared with oe-CircHIPK3 + agomiR-NC group, the apoptosis rate of myocardial tissue in oe-CircHIPK3 + miR-93-5p agomiR group was remarkably decreased (*p* < 0.05) (Figure 4E).

RETRACTED

**Figure 4:** Overexpression of miR-93-5p reverses the myocardial infarction-induced myocardial injury stimulated by CircHIPK3. **(A)** RT-PCR was used to detect the expression of miR-93-5p in myocardial tissue of mice after modeling. **(B)** Pearson's correlation analysis was used to analyze the correlation between miR-93-5p and CircHIPK3. **(C)** 2,3,5-Triphenyltetrazolium chloride staining was used to detect infarct size. **(D)** Masson staining was used to detect collagen deposition. **(E)** TUNEL staining was used to observe the apoptosis of myocardial tissue, *n* = 10. **(F)** RT-qPCR detected miR-93-5p expression in cardiomyocytes *in vitro*. **(G)** The apoptosis of cardiomyocytes was detected by TUNEL staining. **(H)** Western blot analysis detected the expression of Bax, cleaved caspase-3, and Bcl-2 protein. The value in the figures is the measurement data, which is expressed as mean ± standard deviation. The comparison between two groups was analyzed by independent-sample *t*-test. The correlation of circHIPK3 and miR-93-5p was analyzed using Pearson's correlation analysis. The comparison among multiple groups was analyzed by one-way ANOVA, followed by Tukey's multiple-comparisons test. *compared with oe-NC + agomiR-NC group, *p* < 0.05; ^#^compared with oe-CircHIPK3 + agomiR-NC group, *p* < 0.05; ^&^compared with oe-NC + mimic-NC group, *p* < 0.05; ^@^compared with oe-CircHIPK3 + mimic-NC group, *p* < 0.05; ^¥^ compared with control group, *p* < 0.05. The experiment was repeated three times.

RT-qPCR detected miR-93-5p expression in MI cell model *in vitro*. miR-93-5p expression in hypoxia group was significantly lower than that in control group (all *p* < 0.05) (Figure 4F); meanwhile, we set oe-NC + mimic NC group, oe-CircHIPK3 + mimic NC group, and oe-CircHIPK3 + miR-93-5p cotransfection groups. *Versus* the oe-NC + mimic NC group, the apoptosis rate in oe-CircHIPK3 + mimic NC group was clearly increased, while that of oe-CircHIPK3 + miR-93-5p mimic group was lower than that of oe-CircHIPK3 + mimic NC group (all *p* < 0.05) (Figure 4G). The expression of Bax and cleaved caspase-3 was markedly decreased, and Bcl-2 expression was increased after overexpression of circHIPK3 and miR-93-5p (all *p* < 0.05) (Figure 4H). All in all, overexpression of miR-93-5p may inhibit circHIPK3-stimulated myocardial injury.

RETRACTED

### CircHIPK3 Sponges miR-93-5p to Activate the Rac1/PI3K/AKT Pathway

The RNA22 website (https://cm.jefferson.edu/rna22/Precomputed/) found a targeted binding site between miR-93-5p and Rac1 (Figure 5A). Dual-luciferase reporter gene assay showed that miR-93-5p could specifically bind to Rac1 (Figure 5B) (all *p* < 0.05). According to the previous literatures, overexpression of Rac1 can aggravate cardiomyocyte injury during myocardial I/R (27). Therefore, we speculated that circHIPK3 may absorb miR-93-5p, thus upregulating Rac1 expression and participating in myocardial injury after MI. We detected Rac1 expression in myocardial tissue of mice with MI. Relative to the sham group, Rac1 expression in myocardial tissue of MI group was higher than that of the control group (*P* < 0.05); Rac1 expression in MI cell model was higher than that in the control group (Figure 5C). Compared with oe-CircHIPK3 + mimic NC group, overexpression of miR-93-5p and CircHIPK3 in cells suppressed circHIPK3 and Rac1 expression and promoted miR-93-5p expression (all *p* < 0.05); compared with miR-93-5p inhibitor + sh-NC group, miR-93-5p inhibitor + sh-Rac1 group did not affect circHIPK3 and miR-93-5p but decreased Rac1 expression (all *p* < 0.05) (Figure 5D).

**Figure 5:** CircHIPK3 sponges miR-93-5p to activate the Rac1/PI3K/AKT pathway. **(A)** The website predicted the targeting relationship between miR-93-5p and Rac1. **(B)** Dual-luciferase assay was used to verify the targeting relationship between miR-93-5p and Rac1. **(C)** RT-qPCR was used to detect the expression of Rac1 in MI model *in vitro* and *in vivo*. **(D)** RT-qPCR was used to detect the levels of CircHIPK3, miR-93-5p, and Rac1. **(E)** Western blot analysis was used to detect the protein levels of p-PI3K and p-AKT. The value in the figures is the measurement data, which is expressed as mean ± standard deviation. The comparison between two groups was analyzed by independent-sample *t*-test. The comparison among multiple groups was analyzed by one-way ANOVA, followed by Tukey's multiple-comparisons test. *p < 0.05; ^#^*p* < 0.05; ^&^*p* < 0.05. The experiment was repeated three times.

Then, we turned to explore the downstream effectors of Rac1. Rac1 can significantly activate the PI3K/AKT pathway (28–31), and PI3K/AKT pathway activation is related to myocardial injury (32, 33). Therefore, we carried out Western blot analysis to detect the protein levels of p-PI3K and p-AKT. Compared with oe-CircHIPK3 + mimic NC group, overexpression of miR-93-5p and circHIPK3 inhibited the levels of p-PI3K/PI3K and p-AKT/AKT (both *p* < 0.05); compared with miR-93-5p inhibitor + sh-NC group, the levels of p-PI3K and p-AKT in miR-93-5p inhibitor + sh-Rac1 group decreased (all *p* < 0.05) (Figure 5E). Taken together, circHIPK3 absorbed miR-93-5p, thus promoting the activation of the Rac1/PI3K/AKT pathway.

RETRACTED

## Discussion

We performed a series of experiments to verify the underlying circRNA–miR–mRNA network involving circHIPK3 in MI. As expected, we highlighted that circHIPK3 as a ceRNA absorbed miR-93-5p and activated the Rac1/PI3K/AKT pathway. Interference with circHIPK3 upregulated miR-93-5p and then inactivated the Rac1/PI3K/Akt pathway, thus improving MI-induced cardiac dysfunction.

In the past few years, growing evidence has supported the potential role of circRNAs in the pathophysiological process of MI (34–36). We revealed that circHIPK3 expression in myocardial tissue of MI mice and *in vitro* cell model was significantly increased. CircHIPK3 is also highly expressed in cardiomyocytes with simulated myocardial I/R (16). Then, we silenced circHIPK3 expression to examine its effects on MI mice and hypoxia-induced cardiomyocyte injury. Interference with circHIPK3 in MI mice significantly reduced infarct size, collagen deposition, and the rate of myocardial apoptosis. The expression of Bax and cleaved caspase-3 was clearly decreased, and Bcl-2 expression was increased in cardiomyocytes in the hypoxia + sh-CircHIPK3 group. CircHIPK3 silencing attenuates bleomycin-induced collagen deposition in mice with pulmonary fibrosis (37). Blocked proliferation and promoted apoptosis are observed in cardiomyocytes overexpressing circHIPK3 (16). Taken together, circHIPK3 downregulation can reduce cardiomyocyte apoptosis after MI and improve cardiac function.

Current studies have shown that circRNAs possess the ability to bind to miRs *via* acting as molecular sponges (38) and that circRNAs and miRs are closely related in acute MI (39). CircHIPK3 aggravates myocardial I/R injury by sponging miR-124-3p as ceRNA (16). Exosomal circHIPK3 secreted from hypoxia-pretreated cardiomyocytes affects oxidative damage in cardiac microvascular endothelial cells by sponging and modulating the miR-29a/IGF-1 axis (17). CircHIPK3 inhibition sponges miR-29b-3p to prevent angiotensin II-induced cardiac fibrosis (40). We initially unveiled that circHIPK3 could work as a ceRNA to absorb miR-93-5p. Then, we turned to identify miR-93 function in MI. Pearson's correlation analysis discovered that miR-93-5p expression was negatively correlated with circHIPK3. Levels of miR-93 are lower in plasma of MI patients compared with healthy controls (41). The infarct area, collagen deposition, and apoptosis rate in the group overexpressing circHIPK3 and miR-93-5p were significantly decreased. miR-93 elevation after MI is cardiac protective (42). Interestingly, treatment with miR-93-5p-containing exosomes attenuates acute MI-induced myocardial damage (43). Similarly, miR-93 overexpression partially reduces the enhancing effects of MORT overexpression on cardiomyocyte apoptosis (41). Overall, overexpression of miR-93-5p reverses the MI-induced myocardial injury stimulated by circHIPK3.

RETRACTED

Furthermore, we identified the downstream gene and pathway of miR-93-5p in MI. Dual-luciferase assay showed that miR-93-5p could specifically bind to Rac1. Rac-1 is a new therapeutic target in cerebro- and cardio-vascular diseases (44). Rac1 expression is upregulated in myocardial tissue of MI mice and in MI cell model in this study. Cardiac-specific deletion of Rac1 relieves I/R injury in diabetic hearts, whereas cardiomyocytes overexpressing Rac1 predisposes the heart to increased myocardial injury with enhanced contractile dysfunction (45). Knockout of Rac1 in cardiomyocytes partially protects against doxorubicin-induced cardiac injury (27). Rac1 participated in the pathological processes of different brain areas such as ischemic stroke, cognitive disorder, subarachnoid hemorrhage, and representative neuronal oxidative damage of several neurodegenerative disorders (44). Meanwhile, Rac1 may result in the generation of reactive oxygen species by activating nicotinamide adenine dinucleotide phosphate oxidase and thus aggravated cardiomyocyte injury (45, 46). Moreover, Rac1 can activate the PI3K/AKT pathway (31, 47), and activation of the PI3K/AKT pathway is closely related to myocardial injury and even exacerbates cardiomyocyte injury (33, 48). Through Western blot analysis, we highlighted that overexpression of circHIPK3 and miR-93-5p or downregulation of miR-93-5p and Rac1 inhibited the levels of p-PI3K/PI3K and p-AKT/AKT. AKT phosphorylation is increased in infarcted myocardial tissue, and abnormal activation of the PI3K/AKT pathway is related to MI (33). In brief, circHIPK3 can sponge miR-93-5p and activate the Rac1/PI3K/AKT pathway.

In summary, circHIPK3 worked as a ceRNA to absorb miR-93-5p and activate the Rac1/PI3K/AKT pathway. Silencing circHIPK3 upregulated miR-93-5p and inactivated the Rac1/PI3K/Akt pathway, thus improving MI-induced cardiac dysfunction. These results discovered a novel theoretical option for MI treatment. This is still just a preclinical research; although our findings provide therapeutic implications in MI treatment, the experiment results and effective application into clinical practice need further validation. In the future, whether circHIPK3 and miR-93-5p can be biomarkers for early screening of MI remains to be studied. More attention will be paid to study the regulation mechanism of circHIPK3 to seek reliable therapies for MI from the perspective of epigenetics.

RETRACTED

## Data Availability Statement

The original contributions presented in the study are included in the article/supplementary material, further inquiries can be directed to the corresponding author/s.

## Ethics Statement

The animal study was reviewed and approved by Central South University (Changsha).

## Author Contributions

YW and MF were the guarantor of the integrity of the entire study. YW contributed to study design and manuscript editing. MF contributed to study concepts and manuscript preparation. MiW contributed to experimental studies. MiW and JY contributed to the definition of intellectual content. YL and JY contributed to literature research. CY contributed to clinical studies. WP and MeW contributed to data acquisition and data analysis. YL and MiW contributed to statistical analysis. YW, MF, MiW, and CY contributed to manuscript review. All authors read and approved the final manuscript.

## Conflict of Interest

The authors declare that the research was conducted in the absence of any commercial or financial relationships that could be construed as a potential conflict of interest.
